The article "An Attention Mechanism Oriented Hybrid CNN-RNN Deep Learning Architecture of Container Terminal Liner Handling Conditions Prediction" was published in 2021. Journal: Comput Intell Neurosci.

# An Attention Mechanism Oriented Hybrid CNN-RNN Deep Learning Architecture of Container Terminal Liner Handling Conditions Prediction

**DOI:** 10.1155/2021/3846078

**Published:** 2021-07-08

**Authors:** Bin Li, Yuqing He

**Affiliations:** ^1^School of Mechanical and Automotive Engineering, Fujian University of Technology, Fuzhou 350118, China; ^2^School of Transportation, Fujian University of Technology, Fuzhou 350118, China

## Abstract

The booming computational thinking and deep learning make it possible to construct agile, efficient, and robust deep learning-driven decision-making support engine for the operation of container terminal handling systems (CTHSs). Within the conceptual framework of computational logistics, an attention mechanism oriented hybrid convolutional neural network and recurrent neural network deep learning architecture (AMO-HCR-DLA) is proposed technically to predict the container terminal liner handling conditions that mainly include liner handling time (LHT) and total working time of quay crane farm (TWT-QCF) for a calling liner. Consequently, the container terminal oriented logistics generalized computation (CTO-LGC) automation and intelligence are established tentatively by AMO-HCR-DLA. A typical regional container terminal hub of China is selected to design, implement, execute, and evaluate the AMO-HCR-DLA with the actual production data. In the case of severe vibration of LHT and TWT-QCF, while forecasting the handling conditions of 210 ships based on the CTO-LGC running log of four years, the forecasting error of LHT within one hour is more than 97% and that of TWT-QCF within six hours accounts for 89.405%. When predicting the operating conditions of 300 liners by the log of five years, the forecasting deviation of LHT within one hour is more than striking 99% and that of TWT-QCF within six hours reaches up to 94.010% as well. All are far superior to the predicting outcomes by the classical algorithms of machine learning and deep learning. Hence, the AMO-HCR-DLA shows excellent performance for the prediction of CTHS with the low and stable computational consuming. It also demonstrates the feasibility, credibility, and realizability of the computing architecture and design paradigm of AMO-HCR-DLA preliminarily.

## 1. Introduction

For the last decade, deep learning has obtained vigorous development based on the promotion of big data, computing capacity, artificial neural network (ANN), and deep neural network (DNN), especially in the field of computer vision [1–3], image classification [4, 5], speech recognition [6, 7], natural language processing [8, 9], clinical decision support [10, 11], smart manufacturing [12, 13], and so on. In recent years, deep learning is gradually penetrating into the domains of e-commerce and intelligent logistics [14, 15], and it shows a good application prospect.

The article "An Attention Mechanism Oriented Hybrid CNN-RNN Deep Learning Architecture of Container Terminal Liner Handling Conditions Prediction" was published in 2021. Journal: Comput Intell Neurosci.

The container terminals are the backbone and branch hubs of the global transportation network and modern intelligent logistics, which make a crucial effect on the operation and improvement of e-commerce and supply chain all over the world [16]. The container terminal handling systems (CTHS) are the typical representation of complex logistics systems (CLS), and its job planning, task scheduling, and resource allocation all are of representative nondeterministic polynomial complete problems [17]. Those are the big challenges for the traditional methods of operations research, such as mathematical programming [18], intelligent optimization [19], and system simulation [20]. In consequence, the deep learning is gradually applied to the production scheduling and service decision-making of CTHS.

So specifically, the application of deep learning at container terminals can be further subdivided into two categories. One is the traditional application of deep learning for the scenario of container terminals, such as text recognition [21, 22] and object detection [23, 24]. Another is the deep learning for the scheduling and decision support in CTHS [25], such as container relocation problem [26] and container premarshalling problem [27]. The research on the latter is just beginning, which is also the focus of this paper. The agile, efficient, and robust self-evolution, self-learning, and self-adaptive architecture, mechanism, and paradigm in deep learning, which includes recurrent neural network (RNN), convolutional neural network (CNN), and attention mechanism, are expected to supply the new solution to the running of CTHS and improvement of the operational performance of container terminals.

As a result, an attention mechanism oriented hybrid CNN-RNN deep learning architecture (AMO-HCR-DLA) is proposed tentatively to predict the container terminal liner handling conditions that mainly include two aspects: liner handling time (LHT) and total working time of quay crane farm for a calling liner (TWT-QCF). Both are expected to establish a service target time-consuming baseline preliminary sketch for the guidance of the job planning, task scheduling, and resource allocation at container terminals. This is very important for the precise control, efficient operation, and robust execution of CTHS.

The reminder of this paper is organized as follows: Section 2 presents the combination and integration of deep learning and computational logistics by revolving around the calling container liners.  Section 3 proposes AMO-HCR-DLA at length to support the container terminal-oriented logistics generalized computation (CTO-LGC) automation and intelligence. A real case study of CTHS, which covers LHT and TWT-QCF forecasting experiments, performance evaluation, and contrastive analysis by the classical algorithms of machine learning and deep learning together with AMO-HCR-DLA, is fully explored in Section 4.  Section 5 concludes the paper with some discussions and brings forward the directions for future research.

The article "An Attention Mechanism Oriented Hybrid CNN-RNN Deep Learning Architecture of Container Terminal Liner Handling Conditions Prediction" was published in 2021. Journal: Comput Intell Neurosci.

## 2. Deep Learning for Container Terminal Handling Systems by the Combination of Computational Logistics

### 2.1. Computational Logistics for Container Terminal Handling Systems

After ten years of efforts and exploration, the computational logistics was proposed tentatively on the 54th IEEE Conference on Decision and Control in December 2015 [28]. The computational logistics is a unique theoretical approach, engineering solution, design paradigm, algorithm definition, and evaluation compass for programming, planning, scheduling, and decision of CLS to overcome the hierarchy, dynamic, timeliness, nonlinearity, coupling, and complexity (HDT-NCC) that exist widely in CLS.

The CTHS has always been the major research target and carrier in the formation and evolution of computational logistics over the last 15 years [29, 30]. The CTO-LGC is the cornerstone of abstraction and automation for CTHS within the conceptual framework of computational logistics, which is clearly defined according to the essence and connotation of computation [31]. Furthermore, the problem-oriented computability and generalized computational complexity of CTO-LGC both have also been discussed adequately and defined clearly in our previous studies [32, 33], which provide the important theoretical foundations for CTO-LGC from the perspective of the classical theory of computation.

Meanwhile, the hierarchical, parallel, heterogeneous, and reconfigurable computational model of CTHS is proposed by computational logistics which establishes the running architecture of CTO-LGC, and it sets up the efficient and scalable engineering solution to CTO-LGC from the dimension of computational principles [34]. So specifically, the CTO-LGC is implemented and performed by the diversified physical logistics service facilities and equipments, which can be abstracted as the various container logistics generalized computing engine farms. Those mainly cover quay crane (QC), yard crane (YC), internal yard trailer (IYT), container reach stacker (CRS), empty container fork lift (ECFL), container gate house (CGH), and external container truck (ECT). It is evident that the organization, architecture, configuration, deployment, and execution of container logistics generalized computing engine farms have a great contribution to the operational performance of CTHS.

The article "An Attention Mechanism Oriented Hybrid CNN-RNN Deep Learning Architecture of Container Terminal Liner Handling Conditions Prediction" was published in 2021. Journal: Comput Intell Neurosci.

### 2.2. Container Terminal Logistics Generalized Computing Engine Farms Microarchitecture

By computational logistics, the operation of CTHS is highly similar to the running of computer systems whether from the perspective of the system components or in terms of the insights into the operating principles, even at the theoretical level of computation [29, 33]. In consequence, the container terminal oriented logistics generalized computing engine farms microarchitecture (CTO-LGC-EFM) makes a crucial effect on the design, implementation, planning, scheduling, execution, upgrading, and reconstruction of CTHS.

The integral CTHS can be abstracted as a heterogeneous multiprocessor system-on-chip (HMP-SoC) for CTO-LGC that is cast to the plane layout of container terminal. It is the most fundamental definition of CTO-LGC-EFM. Whether the QC is located on quayside or the YC, CRS, or ECFL exists in storage yard all can be abstracted as the CTO-LGC heterogeneous processing units, and then those are connected to implement and fulfill the function of the container accessing, routing, and switching by the unit logistics transmission network for CTO-LGC on HMP-SoC. Furthermore, the CTO-LGC network on chip is also heterogeneous because it is distinctly different at quayside and storage yard. Even all in the storage yard, those have a great deal of differences in the diverse blocks of different properties. In addition, both HMP-SoC and CTO-LGC network on chip are dynamic, parallel, and reconfigurable in practice according to the adjustment of real-time working load and operational ship routes.

Then, the QC, YC, CRS, and ECFL all are the CTO-LGC engine, and those constitute the parallel, heterogeneous, and reconfigurable CTO-LGC physical engine farms, which are just about server clusters for CTO-LGC. In fact, the QC, YC, CRS, and ECFL construct a hybrid CTO-LGC architecture, which is very similar to the collaborative computing architecture of central processing unit (CPU), general purpose graphics processing unit (GPGPU), and synergistic processing element (SPE) in computer science and engineering. It is the combination of serial and parallel and is the hybrid of asynchronous and synchronous as well. More importantly, it is a standard logistics unit accessing and switching network-on-chip in a generalized and distributed computing environment.

According to the status and function of the CTO-LGC diverse physical engines in CTHS, we make a detailed definition of the CTO-LGC physical engine farm. Above all, the QC deserves logistics generalized computation central processing unit (LGC-CPU) of CTHS because it occupies a central position in the operation of CTO-LGC. The LGC-CPU is the container accessing and switching engine between container ships and terminal hubs and is responsible for the loading and discharging container along quay side. It is similar to the CPU in the computer systems, and the LGC-CPU is the most important processing element as well. Furthermore, LGC-CPU can be subdivided into the strong element and the weak one. The former is arterial QC for container trunk liners, and the latter is feeder QC for container feeder vessel. The management of LGC-CPU is mainly involved in QC assignment and scheduling, vessel stowage plan, discharging sequence plan, and loading sequence plan. At the same time, the operation of LGC-CPU has a tremendous impact on the berth allocation plan, internal yard trailer scheduling and YC assignment and scheduling. Therefore, it can be seen that the CTHS possesses high operational dynamics, coupling, uncertainty, and complexity even if only from the point of view.

The article "An Attention Mechanism Oriented Hybrid CNN-RNN Deep Learning Architecture of Container Terminal Liner Handling Conditions Prediction" was published in 2021. Journal: Comput Intell Neurosci.

In the second place, the YC is equivalent to logistics generalized computation general purpose access processing unit (LGC-GPAPU) of CTHS. The YC constitutes an essential component for any storage yard. The YC usually participates in various activities of storage yard actively, such as loading and unloading IYT, stacking, relocation, reshuffle, and premarshalling. As a result, the LGC-GPAPU is considered to have wide versatility. Analogously, the management of LGC-GPAPU is primarily concerned with YC assignment and scheduling, yard allotment plan, yard relocation scheduling, and yard premarshalling plan. Moreover, the execution of LGC-GPAPU has an important influence on the QC assignment and scheduling, CRS scheduling and ECFL dispatching, CGH management, and ECT appointment coscheduling. Thus, the YC assignment and scheduling are the same as that of QC and shows the strong dynamics, coupling, uncertainty, and complexity as well.

Thirdly, the CRS is a kind of mobile machinery, which is considerably different from QC and YC. The CRS is the crucial complement for the operation of storage yard except for YC, and it is identified with logistics generalized computation synergistic processing element (LGC-SPE). The CRS is usually appropriate for a handful of full containers. Generally, the CRS is applied to the sorting and picking containers for a specific purpose. In the same manner, the management of LGC-SPE primarily involves in the CRS scheduling, YC assignment and scheduling, ECFL dispatching, CGH management, and ECT appointment coscheduling.

The article "An Attention Mechanism Oriented Hybrid CNN-RNN Deep Learning Architecture of Container Terminal Liner Handling Conditions Prediction" was published in 2021. Journal: Comput Intell Neurosci.

Last but not least, the ECFL is another kind of mobile machinery and is generally special for the empty container. The ECFL is also an effective supplement for the operation of storage yard except for YC and CRS. Accordingly, the ECFL is optional LGC-SPE for CTHS. Usually, there are a mass of empty containers in the storage yard, especially in China; hence, ECFL may be the more important coprocessor in CTHS compared to CRS.

The above LGC-CPU, LGC-GPAPU, and LGC-SPE all are casting into the terminal plane layout to form the stereolithography lithographic imagery of CTO-LGC physical engine farm to execute container logistics services. Thereupon, the CTO-LGC-EFM can be illustrated by Figure 1, which demonstrates the running of CTO-LGC under typical handling technology and equipment configurations. That shows the CTO-LGC hierarchical structure, switching fabric, and executing framework essentially, and it is critical and crucial to the sound, efficient and error-free operation of CTHS. Apparently, the running performance of LGC-CPU farm is of great significance to the practical operations of CTHS, which can be clearly measured by two indicators of LHT and TWT-QCF. Thereupon, the prediction and evaluation of LHT and TWT-QCF are crucial to the production planning, task scheduling, and resource allocation of CTHS.

### 2.3. Deep Learning for Logistics Generalized Computation Physical Engine Farms

The above CTO-LGC-EFM is the essential conceptual architecture of CTHS for the design and implementation of abstraction and automation by computational logistics. We have expounded the necessity, feasibility, and advancement of combining computational logistics and deep learning in previous studies [35, 36]. Therefore, the deep learning is going to provide the intelligent decision support engine for the scheduling, control, and execution of CTO-LGC-EFM.

According to the above CTO-LGC-EFM, it is concluded that the container liner handling conditions are largely decided by the running and synergy of the LGC-CPU farms. The dynamic load balancing and intelligent allocation scheduling of the LGC-CPU is of great importance to the execution of CTO-LGC. At the same time, both of LHT and TWT-QCF are the most direct manifestation of LGC-CPU farm operation; moreover, the two exert a tremendous influence on the planning and scheduling of LGC-CPU. In fact, the dispatching and allocation of LGC-GPAPU and LGC-SPE are also decided by both to a large extent and even the berth allocation is greatly affected by both. The LHT evaluates liner own operation from the perspective of the carrier, and the TWT-QCF assesses the operational situations of calling ships from the viewing angle of the terminal.

The article "An Attention Mechanism Oriented Hybrid CNN-RNN Deep Learning Architecture of Container Terminal Liner Handling Conditions Prediction" was published in 2021. Journal: Comput Intell Neurosci.

Now, we define and design the AMO-HCR-DLA to forecast the LHT and TWT-QCF, which is supposed to offer an available high-quality reference and guidance for berth allocation, LGC-CPU, LGC-GPAPU, and LGC-SPE assignment and scheduling, especially for the former two. In fact, the berth allocation and the assignment and scheduling of LGC-CPU determine the basic job sequence of the service task process of CTO-LGC. Moreover, the preemption is usually not possible in the berth scheduler, but the LGC-CPU preemption is feasible and frequent during the CTO-LGC. The above CTO-LGC rules affect two operational indicators of LHT and TWT-QCF in turn.

## 3. An Attention Mechanism Oriented Hybrid CNN-RNN Deep Learning Architecture

### 3.1. Core Architecture and Essential Mechanism

The temporal data classification and prediction have been the typical application of machine learning and deep learning [37, 38]. Nicolas et al. [39] applied standard DNN to classify univariate time series generated by discrete and continuous dynamical systems based on their chaotic or nonchaotic behaviors. Fischer and Krauss [40] deployed long short-term memory (LSTM) networks for predicting out-of-sample directional movements for the constituent stocks. Sushil et al. [41] proposed a novel forecasting method that combined LSTM networks and random forest to model complex relationships of both temporal and regression type.

More importantly, both CNN and RNN are applied to the temporal data forecasting in the field of transportation and logistics inch by inch for the past few years. Guerrero-Ibanez et al. [42] discussed some of the challenges that need to be solved to achieve seamless integration between intelligent transportation systems and deep learning methods. Du et al. [43] proposed a dynamic transition CNN for the purpose of precise traffic demand prediction. A novel deep belief network method was employed to mine the inner patterns of flight delays by Yu et al. [44]. Guo et al. [45] designed a perceptron neural network model and proposed to use the deep learning training mechanism to improve the multilayer perceptron neural network, which provided effective technical support for the improvement of the model of predicting the demand for industrial logistics. As the hinge between water-transportation and land-carriage, deep learning is also gradually applied to the container terminal operations [46]. Especially, RNN and CNN are frequently used in the throughput prediction of container terminals [47–50]. Nevertheless, the prediction of LHT and TWT-QCF is relatively rare at the tactical and execution levels because both are of more sophisticated level of analysis and prediction.

The article "An Attention Mechanism Oriented Hybrid CNN-RNN Deep Learning Architecture of Container Terminal Liner Handling Conditions Prediction" was published in 2021. Journal: Comput Intell Neurosci.

Therefore, we introduce a new principle into the algorithm that is an attention mechanism. The attention mechanism has been widely applied in the image segmentation [51], object detection [52], speech recognition [53], machine translation [54], mass customization [55], chaotic time series forecasting [56], and so on. However, there are few examples of attention mechanism being applied to the management of CLS, let alone to operational decisions at container terminals. In conclusion, we integrate RNN, CNN, and attention mechanism to propose AMO-HCR-DLA for the prediction of container terminal liner handling conditions. It is a beneficial attempt for the exploration and application of deep learning in CLS within the conceptual framework of computational logistics.

### 3.2. Attention Mechanism Oriented Hybrid Computing Architecture

Compared with the prediction of liner berthing time (LBT), the liner handling conditions are more difficult to forecast because the factors and uncertainties involved are more complicated and the granularity of analysis and prediction is finer. Furthermore, the AMO-HCR-DLA is expected to be appropriate for the prediction of LHT and TWT-QCF simultaneously. According to the multiple container terminal production instances, the number of layers in AMO-HCR-DLA usually reaches 10 to 20, which is the typical DNN learning architecture. Accordingly, the attention mechanism oriented CNN-RNN multilayer hybrid computing architecture is demonstrated by Figure 2 in a capsule.

The AMO-HCR-DLA is a typical lightweight computing architecture, and it includes multiple key components that are executed in sequence. The AMO-HCR-DLA does not require much hardware, but is extremely suitable for GPU parallel computing architecture, especially for the module of deep learning model. It makes the AMO-HCR-DLA possess extremely high computational efficiency and response agility, and the computing time of AMO-HCR-DLA is usually only a few minutes.

Specifically speaking, the AMO-HCR-DLA is a typical functional model, and it mainly consists of five components that are deep learning engine preheating, operational log data preprocessing, CTO-LGC execution deep learning model, ANN model evaluation of terminal logistics service, and liner handling conditions prediction outcome for intelligent decision support, respectively. The most core component is apparently deep learning model that is a representative hybrid ANN computing architecture. Now, we discuss the theme in detail.

### 3.3. Kernel Processes and Computing Paradigm

With respect to our previous discussion on the prediction of LBT [36], the prediction of LHT and TWT-QCF is much more difficult because of the value range and vibration degree. Accordingly, two core elements of the DNN model can be summarized below. One of the crucial steps is the combination of RNN and CNN to dramatically increase performance of the ANN model. The AMO-HCR-DLA includes RNN that covers LSTM, gated recurrent unit (GRU), bidirectional-LSTM, and bidirectional-GRU, CNN, dense network, dropout layer, noise layer, advanced activation layer, self-defining layers, and so on. Another important point is the definition of the attention mechanism module on the input dimensions, which aims at compelling the model to pay more attention to the decisive feature dimensions and relatively ignore other feature dimensions. It is evident that the AMO-HCR-DLA is tailorable, configurable, tunable, and customized, which is crucial and critical for the agility, flexibility, and portability of the DNN learning model for CTHS.

The article "An Attention Mechanism Oriented Hybrid CNN-RNN Deep Learning Architecture of Container Terminal Liner Handling Conditions Prediction" was published in 2021. Journal: Comput Intell Neurosci.

More importantly, for deep learning model core computing architecture of LBT forecasting in our previous discussion, the Python package, very time series feature extraction on basis of scalable hypothesis tests named as tsfresh [57], makes a crucial effect on the improvement of DNN model performance [36]. The tsfresh has a low computational complexity and a wide range of application fields [58, 59]. Nevertheless, the tsfresh needs manual intervention to filtrate the statistical characteristics in the phase of data preprocessing. It is a repeated attempt and time-consuming work. The combination of CNN and attention mechanism takes the place of tsfresh to eliminate the measure and defect with an adaptive and efficient computing paradigm and obtains the outstanding self-adaptation and self-learning performance that is shown in Figure 3. Those are the kernel processes and computing paradigm of AMO-HCR-DLA substantially which yields dramatic increases in the agility, flexibility, robustness, and portability for DNN model too.

Specifically speaking, the RNN layers are the main core architecture of forecasting. Meanwhile, both CNN layers and attentional mechanism have the property of emphasizing some weights for CTO-LGC feature vector. The former is in front of RNN layers, and the latter is behind of the combination of LSTM and GRU, which helps RNN layers to obtain better forecasting behavior. Looking from the other side, the RNN encodes into the time dependency of CTO-LGC log, the CNN encodes into the space dependency of CTO-LGC log, and the attention mechanism adaptively adjusts the proportion of temporal and spatial coupling factors that are represented by the feature vector of CTO-LGC. As a matter of fact, it is the design philosophy of the AMO-HCR-DLA.

## 4. Deep Learning Computational Experiments for Container Terminal Logistics Service

### 4.1. Case Scenario and Loading Job Set Analysis

A regional and traditional container terminal hub in China is the target object for the demonstration of the AMO-HCR-DLA. There are five deep water berths along terminal quayside, and ten quay cranes with the four different activation parameters and handling specifications are deployed along terminal quayside. The annual container throughput of terminal is about two million twenty-foot equivalent units (TEUs). About 75 to 85 percent of the visiting container ships is attached to the domestic trade routes in China as appropriate, and the other liners serve for international trade routes. It is a very typical large-scale container terminal hub by the east coast of China.

The article "An Attention Mechanism Oriented Hybrid CNN-RNN Deep Learning Architecture of Container Terminal Liner Handling Conditions Prediction" was published in 2021. Journal: Comput Intell Neurosci.

We focus on the domestic trade liners to discuss the AMO-HCR-DLA because those occupy the main parts of the terminal service object. We select the data set of calling liners for 5 years in a row to carry out the machine learning and deep learning computational experiments. Although all are domestic trade ships, both of LHT and TWT-QCF are still terribly different among the liners, which can be obtained from Figures 4 and 5 , Tables 1 and 2 together. To all appearances, the Pearson correlation coefficient of between LHT and TWT-QCF is 0.788, and the two-tailed significance is 0.000. It seems that the two are highly interrelated, and the relevant quadratic fit line is shown in Figure 6. However, the TWT-QCF is not necessarily greater than the LHT; furthermore, there is not a clear decisive relationship between LHT and TWT-QCF. All make it extremely difficult to predict LHT and TWT-QCF with one model.

According to the above Tables 1 and 2, it is concluded that the size of the target data set is 9433 items, which is a very classical small data set whether for machine learning or for deep learning in effect. It is important to point out that the liners whose LHT is within 20 hours come up to 95.897% of the total, and the ships whose LHT is within 25 hours go as high as 99.237%, and the vessels whose LHT is within 30 hours reach up to amazing 99.830%. It means that the log records whose LHT is over 25 hours all can be considered as the stochastic disturbance noise during the machine learning and deep learning computational process. Based on Table 2 and Figure 5, it is reasonable to infer that the variation range of TWT-QCF is far greater than the one of LHT. It should also be noted that the liners whose TWT-QCF is within 60 hours come up to 97.880% of the total, the ships whose TWT-QCF is within 80 hours go as high as 99.205%, and the vessels whose TWT-QCF is within 100 hours also reach up to 99.830%. It is also a sign that the log records whose TWT-QCF is over 60 hours all can be regarded as the stochastic disturbance noise for the machine learning and deep learning too.

The article "An Attention Mechanism Oriented Hybrid CNN-RNN Deep Learning Architecture of Container Terminal Liner Handling Conditions Prediction" was published in 2021. Journal: Comput Intell Neurosci.

Meanwhile, the hardware platform is very common, which is easy to set up and is cost effective. The central processing unit (CPU) is the Intel Core Intel i7-9750H and the graphics processing unit (GPU) is the NVIDIA GeForce GTX 1660 Ti. The main memory is 24 GB, and the video memory is 6 GB. In order to compare and analyze the performance differences among multifarious prediction algorithms, those are executed by the different platforms. The machine learning is designed and implemented by SPSS 25 and MATLAB 2020b which cover two kinds of classical time series prediction analysis algorithms, and the deep learning software platform is primarily based on the TensorFlow 2.3 for GPU.

### 4.2. Calling Liner Handling Conditions Prediction by Machine Learning

Considering that the prediction of LHT and TWT-QCF is very difficult, the CTO-LGC log is executed and evaluated by the classical machine learning algorithms. Above all, we design and execute the cluster analysis of LHT and TWT-QCF by using K-Means method to evaluate the characteristics of the CTO-LGC log, which is implemented by SPSS 25. The selected cluster variables mainly include service route number, shipping company encoding, length of calling vessel, LBT, LHT, TWT-QCF, total handling volume by container units, total handling volume by TEUs, shifting quantity of hatch cover, vessel rate by container units, vessel rate by TEUs, gross crane rate by container units, and gross crane rate by TEUs. All the significances of cluster variables are 0.000 in the analysis of variance. It indicates that those are extremely significant, which means that the selection of cluster variables is sound, valid, and effective. The final cluster centers are shown in Table 3. The CTO-LGC log is divided into five categories whose number is 124, 339, 4671, 853, and 3446 in sequence. The LHTs in the final cluster centers are 24.364, 18.536, 6.291, 15.189, and 11.748, respectively, and the TWT-QCFs in the final cluster centers are 80.777, 53.457, 5.801, 29.905, and 15.155 apart. Even all for the domestic container liners, the differences of LHT and TWT-QCF among them are still very obvious because the clustering centers are far apart distinctly. It demonstrates the difficulty level of LHT and TWT-QCF forecasting from another visual angle.

For one thing, the autoregressive integrated moving average model (ARIMA), which is one of the most classic time series prediction algorithms in the machine learning, is used for the container terminal liner handling conditions predictions. The ARIMA is implemented and executed by SPSS 25 too, and it is applied for the forecasting of LHT and TWT-QCF for 300 calling liners based on CTO-LGC log of five years. The prediction of the algorithm is compared with the actual production results by Figures 7 and 8 apart. To all appearances, the ARIMA has a poor performance for LHT or TWT-QCF, and it is not applicable to the complex situations' prediction for CTHS.

The article "An Attention Mechanism Oriented Hybrid CNN-RNN Deep Learning Architecture of Container Terminal Liner Handling Conditions Prediction" was published in 2021. Journal: Comput Intell Neurosci.

For another, the Fine Gaussian Support Vector Machine (FG-SVM), which is the classical regression analysis algorithm for machine learning too [60], is used to make the prediction of LHT and TWT-QCF for 300 calling liners based on CTO-LGC log of five years. The FG-SVM has been designed and implemented as a component in the application of regression learner in MATLAB 2020b. Through debugging the application of FG-SVM repeatedly, the comparison of LHT and TWT-QCF representative predictors with real values is shown by Figures 9 and 10 . Obviously, the FG-SVM does not work very well whether for LHT or TWT-QCF as well. For the phase of training and validation, the final mean absolute error (MAE) is 1.7403 for LHT by FG-SVM, and the ultimate MAE is 4.4895 for TWT-QCF. Both are also unsatisfactory. As a result, the deep learning is introduced tentatively to forecast the container liner handling conditions.

### 4.3. Calling Liner Handling Conditions Prediction with Deep Learning

In our previous studies, we have utilized deep learning to carry out research on LBT at container terminals [35]. The deep learning model core computing architecture (DLM-CCA), which is clearly defined in [35], is a typical combination of LSTM, GRU, and noise layer, and it obtains a good performance for LBT. By the light of nature, the DLM-CCA is expected to be same with LHT. As a result, the LHT of 300 calling liners is going to be predicted by DLM-CCA on the basis of CTO-LGC log of five years. The typical DLM-CCA training loss curves, which is measured by the MAE, is demonstrated by Figure 11. In the meantime, the contrast between typical LHT forecasting with actual values can be displayed by Figure 12. It is easy to deduce that the DLM-CCA does not meet the prediction requirements of LHT. Thereupon, the AMO-HCR-DLA is executed to forecast LHT.

For verifying and testing the adaptation, self-learning and fitting characteristics of AMO-HCR-DLA, the above CTO-LGC log is distinguished as two data sets. The first data set covers 6597 items, and it is actually the CTO-LGC log of four years, which is called after the liner handling conditions for the four years (LHC-OUR). The second data set includes 9433 records, and it is the CTO-LGC log of five years in effect, which is named after the liner handling conditions for the five years (LHC-IVE).

The article "An Attention Mechanism Oriented Hybrid CNN-RNN Deep Learning Architecture of Container Terminal Liner Handling Conditions Prediction" was published in 2021. Journal: Comput Intell Neurosci.

Both LHC-OUR and LHC-IVE are segmented into three main sections that are training set, validation one, and testing one, and the proportions of the three are 80.000%, 16.820%, and 3.180% apart. Consequently, the LHT of 210 and 300 calling container ships are going to be forecasted about three weeks and a month's worth of visiting liners for China's domestic trade requirements. In other words, the AMO-HCR-DLA can make a decision support for the CTO-LGC planning and scheduling of three weeks and a month in this case, especially for terminal quayside production, which is of great concern for the operation of CTHS at the tactical and execution level. Now, we emphatically expound the design and experiment on the AMO-HCR-DLA for the LHT forecasting.

For the current instances, the AMO-HCR-DLA is a 15-layer DNN structure. Above all, the input layer specifies the shape of the input data of the model. Secondly, a dense full-connection layer is set as the output layer. Lastly, the RNN, CNN, and noise layer constitute the other layers with the attention mechanism, and the number of neurons output in each layer is distinctly different. The activation function of the model covers ReLU, tanh, and Sigmoid, and the optimizer is classical Adam.

Subsequently, for LHC-OUR and LHC-IVE, we perform the AMO-HCR-DLA for 100 times with the different random number seeds separately. The running of AMO-HCR-DLA has excellent reproducibility for the same seed, which is an outstanding quality of AMO-HCR-DLA. The typical DNN model training loss curves based on LHC-OUR and LHC-IVE can be illustrated by Figures 13 and 14 separately. Meanwhile, the contrast between typical LHT forecasting with actual values can be displayed by Figures 15 and 16 . In addition, the prediction deviation profiles of LHT by the AMO-HCR-DLA for LHC-OUR and LHC-IVE are shown by Tables 4 and 5 . All give an initial insight into the deep learning ANN model architecture and parameters.

It is easy to draw the conclusion that the AMO-HCR-DLA supplies the sound, efficient, and robust references for intelligent decision support of CTHS in line with Figures 15 and 16 and Tables 4 and 5. In the case of severe vibration of LHT, for LHC-OUR, the experimental results show that the prediction error within one-hour accounts for more than 97%. The corresponding experimental results based on LHC-IVE is responsible for 99.110 percent. In contrast to AMO-HCR-DLA, the prediction error within one hour only accounts for 12.333% and 55.333% while applying the ARIMA and FG-SVM for LHC-IVE to execute machine learning for LHT, and the prediction error within four hours is just 48.000% and 85.000%. At the same time, the forecast error within one hour and four hours are 17.933% and 64.600% severally by DLM-CCA. All indicate that the AMO-HCR-DLA has excellent learning performance and no overfitting. This will bring great convenience for the planning and scheduling of CTHS. It suggests that the AMO-HCR-DLA can acquire a rational and dependable decision reference of LHT using a feasible, reliable, and efficient mode, which demonstrates good follow-up and credibility.

The article "An Attention Mechanism Oriented Hybrid CNN-RNN Deep Learning Architecture of Container Terminal Liner Handling Conditions Prediction" was published in 2021. Journal: Comput Intell Neurosci.

### 4.4. Total Working Time Forecasting of Quay Crane Farm with Deep Learning

For the same data set and hardware platform, we start a discussion of predictions for TWT-QCF with the same DLM-CCA and AMO-HCR-DLA, and even the parameters are all identical. The only difference is that the feature items need to be adjusted through the drop function due to different prediction targets. In like manner, the TWT-QCF of 300 calling liners is going to be predicted by DLM-CCA on the basis of LHC-IVE. The typical DLM-CCA training loss curves, which is measured by the MAE too, is demonstrated by Figure 17. Meanwhile, the contrast between typical TWT-QCF forecasting with actual values can be displayed by Figure 18. It is easy to deduce that the DLM-CCA does not meet the prediction requirements of TWT-QCF, especially when it shakes violently.

Similarly, we perform the AMO-HCR-DLA for 100 times with the different random number seeds based on LHC-OUR and LHC-IVE, respectively. The training loss curves of typical ANN model based on two data sets can be illustrated separately in Figures 19 and 20 , and the comparisons between typical TWT-QCF forecasting with actual values can be illustrated in Figures 21 and 22 . In the meantime, the prediction deviation profiles of TWT-QCF by the AMO-HCR-DLA are shown by Tables 6 and 7 .

Obviously, the AMO-HCR-DLA supplies the feasible and reasonable references for TWT-QCF. Because the TWT-QCF is more volatile than the LHT, based on LHC-OUR, the proportion of prediction error of TWT-QCF within one hour is 36.329%, while the proportion of prediction error of TWT-QCF within six hours achieves 89.405%. Based on LH-IVE, the prediction error of TWT-QCF within one hour is only 32.087%, but the prediction error of TWT-QCF within six hours reaches up to 94.010%. Given that there are usually multiple QCs handling on a ship simultaneously and that the QC may be joined or withdrawn during the operation, this prediction error is acceptable and favorable. Taking it a step further, for LHC-OUR, the proportion of prediction error of TWT-QCF within ten hours reaches up to 97.038%, and the corresponding proportion achieves 97.103% for LHC-IVE. Both are nearly identical. It can be found that the forecasting error of TWT-QCF is more than 10 times relative to that of LHT based on the corresponding data sets.

The article "An Attention Mechanism Oriented Hybrid CNN-RNN Deep Learning Architecture of Container Terminal Liner Handling Conditions Prediction" was published in 2021. Journal: Comput Intell Neurosci.

As described in Section 4.1, when the TWT-QCF exceeds 70 hours, it is difficult for the machine learning and deep learning to predict the effective solution. Meanwhile, the prediction error within one-hour only accounts for 5.000% and 35.000% while applying the ARIMA and FG-SVM for LHC-IVE to execute machine learning for TWT-QCF, and the prediction error within six hours is just 31.667% and 78.667%, and the prediction error within ten hours is merely 48.667% and 87.667%. As for the DLM-CCA, the prediction error within one-hour, six one, and ten ones are only 9.400%, 51.300%, and 70.400% apart. Consequently, the defect of the AMO-HCR-DLA is acceptable and prominent. Hence, the AMO-HCR-DLA provides a reasonable and reliable prediction values for TWT-QCF in the vast majority of cases.

### 4.5. Deep Learning Performance Evaluation of Liner Handling Conditions

According to Sections 4.3 and 4.4, it is concluded that the AMO-HCR-DLA has excellent and effective performance for the prediction of liner handling conditions. As a matter of fact, the AMO-HCR-DLA reveals sound and robust performance at any stage of deep learning whether for LHT or for TWT-QCF.

On the one hand, the indicator of MAE is applied to assess evolution and learning effects of AMO-HCR-DLA during the process of training and validation. For the indicator of LHT, at the end of ANN model training, the final MAE values of the 100 experiments based on LHC-OUR are between 0.0118 and 0.0134, with an average of 0.0124. The final Mae values of 100 experiments based on LHC-IVE range from 0.0091 to 0.0102, and the average value is 0.0096. In the validation phase of ANN model learning, the final MAE values of 100 experiments with LHC-OUR are between 0.0055 and 0.0132, with an average of 0.0074. The final MAE values of 100 experiments with LHC-IVE are between 0.0040 and 0.0080, and the mean is 0.0054. Those are close to the theoretical optimal value of MAE. In terms of TWT-QCF, at the end of ANN model training, the final MAE values of 100 experiments based on LHC-OUR are between 0.0199 and 0.0217, with an average value of 0.0211. Using LHC-IVE, the final MAE values are between 0.0197 and 0.0218 in 100 experiments, and the average value is 0.0201. In the validation phase of ANN model learning, the final MAE values of 100 experiments with LHC-OUR range from 0.0252 to 0.0276, with an average of 0.0262. The corresponding final MAE values using LHC-IVE range from 0.0220 to 0.0257, and the mean is 0.0226. All of the above are close to the theoretical optimal value of MAE too.

The article "An Attention Mechanism Oriented Hybrid CNN-RNN Deep Learning Architecture of Container Terminal Liner Handling Conditions Prediction" was published in 2021. Journal: Comput Intell Neurosci.

On the other hand, the MAE, root mean squared error (RMSE), coefficient of determination of *R*-square, and explained variance score (EVS) together establish the core evaluation metrics of LHT and TWT-QCF forecasting performance for the testing phase displayed from Tables 8–11 . The theoretical optimal value of the first two is 0, and the latter two is one. Meanwhile, while applying the FG-SVM for LHC-IVE to execute machine learning for LHT, the values of MAE, RMSE, *R*-square, and EVS are 2.06796667, 3.66077355, 0.55797117, and 0.59245178 apart in the testing phase. The values of MAE, RMSE, *R*-square, and EVS are 5.99190000, 14.49682665, 0.42343926, and 0.44556227, respectively, during the testing phase by the FG-SVM for LHC-IVE to execute regression analysis for TWT-QCF.

In addition, when the DLM-CCA is applied to implement deep learning for LHT based on LHC-IVE for ten times experiments, the average values of MAE, RMSE, *R*-square, and EVS in the testing phase are 3.47704540, 4.35120713, 0.37524279, and 0.37691790, respectively. Similarly, the DLM-CCA is executed TWT-QCF forecasting based on LHC-IVE for ten times experiments, the mean of MAE, RMSE, *R*-square, and EVS in the testing phase are 9.68388839, 15.35464391, 0.35289795, and 0.37103933 apart. It is evident that the performance of AMO-HCR-DLA is far superior to that of FG-SVM and DLM-CCA from any of the above indicators.

On those measures, the AMO-HCR-DLA has good performance for LHT and TWT-QCF in an absolute sense, especially for the former. Through the above four indicators, it is also concluded that the forecasting accuracy of LHT is far ahead of the one of TWT-QCF. In particular, the MAE and RMSE of TWT-QCF are almost ten times as high as the two of LHT. Moreover, the standard deviation and variance of the four indicators are close to 0, especially for R-square and EVS. It shows that the LHT and TWT-QCF forecasting performance of the AMO-HCR-DLA is very workable, stable, credible, and reliable, which can provide great convenience for the intelligent decision support to the rolling plan, periodic scheduling, and real-time control at container terminals.

## 5. Conclusions

This paper focuses on the automation and intelligentization of CTO-LGC by the combination, integration, and fusion of computational logistics and deep learning and proposes a feasible, dependable, efficient, and robust deep learning architecture for container terminal liner handling conditions that is exact AMO-HCR-DLA. The AMO-HCR-DLA is the integration and synthesis of RNN, CNN, and attention mechanism whose combination is rarely applied to the forecasting and decision of CLS at the tactical and execution level. Furthermore, the AMO-HCR-DLA can be applied to the prediction and analysis of several key operational indicators simultaneously with a small dataset although it cannot obtain the same prediction accuracy for multiple indicators at present. The AMO-HCR-DLA establishes a sound and reliable decision support foundation for the planning, scheduling, and execution of CTO-LGC, which relies on ANN computing architecture to realize intelligent automation of container terminal logistics service consequently. In the future, the DNN customization philosophies and parameter tuning strategy for AMO-HCR-DLA are going to be further discussed to implement the high precision and low computational cost for the multiple key operational indexes of CTHS, which is not just limited to the indicators of LHT and TWT-QCF.

The article "An Attention Mechanism Oriented Hybrid CNN-RNN Deep Learning Architecture of Container Terminal Liner Handling Conditions Prediction" was published in 2021. Journal: Comput Intell Neurosci.

## Figures and Tables

**Figure 1:** CTO-LGC engine farms microarchitecture based on computational logistics.

**Figure 2:** Attention mechanism oriented CNN-RNN multilayer computing architecture.

**Figure 3:** Kernel processes and computing paradigm of AMO-HCR-DLA.

**Figure 4:** Distribution preliminary sketch of calling liners handling time.

**Figure 5:** Distribution preliminary sketch of total working time of quay crane farm.

**Figure 6:** Correlation analysis between LHT and TWT-QCF for Chinese domestic trade routes.

**Figure 7:** A comparison of LHT representative predictors with real values by ARIMA.

**Figure 8:** A comparison of TWT-QCF representative predictors with real values by ARIMA.

**Figure 9:** A comparison of LHT representative predictors with real values by FG-SVM.

**Figure 10:** A comparison of TWT-QCF representative predictors with real values by FG-SVM.

**Figure 11:** A typical DLM-CCA training loss curve for LHT.

**Figure 12:** A comparison of LHT representative predictors with real values by DLM-CCA.

**Figure 13:** A typical AMO-HCR-DLA training loss curve for LHT with LHC-OUR.

**Figure 14:** A typical AMO-HCR-DLA training loss curve for LHT with LHC-IVE.

**Figure 15:** A comparison of LHT representative predictors with real values for LHC-OUR by AMO-HCR-DLA.

**Figure 16:** A comparison of LHT representative predictors with real values for LHC-IVE by AMO-HCR-DLA.

**Figure 17:** A typical DLM-CCA training loss curve for TWT-QCF.

**Figure 18:** A comparison of TWT-QCF representative predictors with real values by DLM-CCA.

**Figure 19:** A typical AMO-HCR-DLA training loss curve for TWT-QCF with LHC-OUR.

**Figure 20:** A typical AMO-HCR-DLA training loss curve for TWT-QCF with LHC-IVE.

**Figure 21:** A comparison of TWT-QCF representative predictors with real values for LHC-OUR by AMO-HCR-DLA.

The article "An Attention Mechanism Oriented Hybrid CNN-RNN Deep Learning Architecture of Container Terminal Liner Handling Conditions Prediction" was published in 2021. Journal: Comput Intell Neurosci.

**Figure 22:** A comparison of TWT-QCF representative predictors with real values for LHC-IVE by AMO-HCR-DLA.

**Table 1:** Distribution characteristic values of LHT for Chinese domestic trade routes (hours).

Year	Quantity of liners	Minimum of LHT	Maximum of LHT	Mean of LHT	Median of LHT	Mode of LHT	Standard deviation of LHT	Variance of LHT
RA	1422	0.2050	31.6670	8.5949	8.0000	9.3330	4.6534	21.6544
RB	1264	0.1220	24.3300	8.2810	7.8330	9.3330	4.4853	20.1177
RC	1350	0.1870	31.5000	8.7798	8.0830	7.5000	4.8439	23.4636
RD	2561	0.1230	33.2500	10.5207	10.0330	8.5000	5.3946	29.1022
RE	2836	0.2330	39.8330	10.8050	10.2505	11.3330	5.5508	30.8118

**Table 2:** Distribution characteristic values of TWT-QCF for Chinese domestic trade routes (hours).

Year	Quantity of liners	Minimum of TWT-QCF	Maximum of TWT-QCF	Mean of TWT-QCF	Median of TWT-QCF	Mode of TWT-QCF	Standard deviation of TWT-QCF	Variance of TWT-QCF
RA	1422	0.0800	86.2900	11.0011	8.4850	2.1000	10.1738	103.5067
RB	1264	0.0200	68.7700	10.8218	8.7550	1.6200	9.3594	87.5990
RC	1350	0.0700	96.3500	11.9635	8.3600	2.3700	12.3734	153.1003
RD	2561	0.0200	117.6600	15.8854	11.8100	11.1500	15.1554	229.6847
RE	2836	0.1700	129.4800	16.5057	11.8350	8.0300	17.0476	290.6211

**Table 3:** Final cluster centers of CTO-LGC log data set with the five years.

Cluster variables	Cluster 1	Cluster 2	Cluster 3	Cluster 4	Cluster 5
Length of calling vessel	230.689	241.043	101.312	186.309	122.795
Liner berthing time	25.657	20.038	7.886	16.632	13.138
Liner handling time	24.364	18.536	6.291	15.189	11.748
Total working time of quay crane farm	80.777	53.457	5.801	29.905	15.155
Total volume of container units	2281	1450	142	748	365
Total volume of TEUs	2479.355	1596.131	193.334	861.999	464.078
Shifting quantity of hatch cover	47	35	10	20	18
Vessel rate by container units	95.960	80.788	23.569	51.943	33.068
Vessel rate by TEUs	104.217	88.858	33.293	59.809	42.233
Gross crane rate by container units	29.288	28.051	28.089	26.169	25.846
Gross crane rate by TEUs	31.869	30.919	40.200	30.299	33.318

**Table 4:** Prediction deviation profile of liner handling time with LHC-OUR.

Prediction deviation (hours)	Minimum of liners	Maximum of liners	Mean of liners	Median of liners	Mode of liners	SD of liners	Variance of liners	Quantitative proportion of liners (%)
[0, 0.2]	40.0000	144.0000	109.7000	113.5000	114.0000	21.1208	446.0900	52.2381
(0.2, 0.4]	41.0000	90.0000	61.6000	60.0000	59.0000	9.5572	91.3400	29.3333
(0.4, 0.6]	7.0000	54.0000	23.8700	23.0000	19.0000	9.5558	91.3131	11.3667
(0.6, 0.8]	0.0000	50.0000	7.6400	7.0000	7.0000	6.2458	39.0104	3.6381
(0.8, 1.0]	0.0000	10.0000	2.3500	2.0000	2.0000	1.7965	3.2275	1.1190
(1.0, +∞]	2.0000	19.0000	4.8400	5.0000	5.0000	2.0086	4.0344	2.3048

The article "An Attention Mechanism Oriented Hybrid CNN-RNN Deep Learning Architecture of Container Terminal Liner Handling Conditions Prediction" was published in 2021. Journal: Comput Intell Neurosci.

**Table 5:** Prediction deviation profile of liner handling time with LHC-IVE.

Prediction deviation (hours)	Minimum of liners	Maximum of liners	Mean of liners	Median of liners	Mode of liners	Standard deviation of liners	Variance of liners	Quantitative proportion of liners (%)
[0.0, 0.2]	78.0000	225.0000	170.1700	178.5000	133.0000	32.5269	1058.0011	56.7233
(0.2, 0.4]	56.0000	129.0000	85.0700	84.5000	63.0000	15.9080	253.0651	28.3567
(0.4, 0.6]	5.0000	75.0000	29.3600	26.0000	34.0000	13.6474	186.2504	9.7867
(0.6, 0.8]	0.0000	23.0000	9.1200	8.0000	6.0000	5.2655	27.7256	3.0400
(0.8, 1.0]	0.0000	13.0000	3.6100	3.0000	0.0000	2.8806	8.2979	1.2033
(1.0, +∞]	0.0000	18.0000	2.6700	0.5000	0.0000	4.2475	18.0411	0.8900

**Table 6:** Prediction deviation profile of total working time of quay crane farm with LHC-OUR.

Prediction deviation (hours)	Minimum of liners	Maximum of liners	Mean of liners	Median of liners	Mode of liners	SD of liners	Variance of liners	Quantitative proportion of liners (%)
[0.0, 2.0]	109.0000	148.0000	125.4700	125.0000	127.0000	7.3205	53.5891	59.7476
(2.0, 4.0]	27.0000	60.0000	44.0400	44.0000	41.0000	6.8439	46.8384	20.9714
(4.0, 6.0]	9.0000	29.0000	18.2400	18.5000	20.0000	4.2074	17.7024	8.6857
(6,0, 8.0]	5.0000	17.0000	10.7400	11.0000	11.0000	2.5559	6.5324	5.1143
(8.0, 10.0]	0.0000	13.0000	5.2900	5.0000	4.0000	2.6844	7.2059	2.5190
(10.0, +∞]	4.0000	11.0000	6.2200	6.0000	7.0000	1.8198	3.3116	2.9619

**Table 7:** Prediction deviation profile of total working time of quay crane farm with LHC-IVE.

Prediction deviation (hours)	Minimum of liners	Maximum of liners	Mean of liners	Median of liners	Mode of liners	Standard deviation of liners	Variance of liners	Quantitative proportion of liners (%)
[0.0, 2.0]	133.0000	226.0000	188.6400	189.0000	182.0000	16.2798	265.0304	62.8800
(2.0, 4.0]	43.0000	138.0000	74.1800	70.5000	63.0000	17.6779	312.5076	24.7267
(4.0, 6.0]	7.0000	39.0000	19.2100	18.0000	11.0000	7.2032	51.8859	6.4033
(6,0, 8.0]	0.0000	12.0000	5.6300	6.0000	5.0000	2.5364	6.4331	1.8767
(8.0, 10.0]	0.0000	9.0000	3.6500	3.0000	5.0000	2.0561	4.2275	1.2167
(10.0, +∞]	7.0000	28.0000	8.6900	8.0000	7.0000	2.4807	6.1539	2.8967

**Table 8:** Predictive performance evaluation profiles of LHT experiment for the testing phase with LHC-OUR.

Evaluation indicators	Minimum of indicators	Maximum of indicators	Mean of indicators	Median of indicators	Standard deviation of indicators	Variance of indicators
MAE	0.20370305	0.54879972	0.28335165	0.27650864	0.04974772	0.00247484
RMSE	0.37573466	0.77587897	0.52617718	0.52754567	0.05293213	0.00280181
*R*-square	0.98095644	0.99553396	0.99115298	0.99119597	0.00185469	0.00000344
EVS	0.98837441	0.99555821	0.99202271	0.99189429	0.00126606	0.00000160

The article "An Attention Mechanism Oriented Hybrid CNN-RNN Deep Learning Architecture of Container Terminal Liner Handling Conditions Prediction" was published in 2021. Journal: Comput Intell Neurosci.

**Table 9:** Predictive performance evaluation profiles of LHT experiment for the testing phase with LHC-IVE.

Evaluation indicators	Minimum of indicators	Maximum of indicators	Mean of indicators	Median of indicators	Standard deviation of indicators	Variance of indicators
MAE	0.14756905	0.38431970	0.22615878	0.22290859	0.04764056	0.00226962
RMSE	0.18532077	0.51163393	0.29800431	0.28932544	0.06317552	0.00399115
*R*-square	0.99136577	0.99886720	0.99693915	0.99723889	0.00135355	0.00000183
EVS	0.99516424	0.99887164	0.99772628	0.99786399	0.00076309	0.00000058

**Table 10:** Predictive performance evaluation profiles of TWT-QCF experiment for the testing phase with LHC-OUR.

Evaluation indicators	Minimum of indicators	Maximum of indicators	Mean of indicators	Median of indicators	Standard deviation of indicators	Variance of indicators
MAE	2.32481191	3.30981076	2.73152114	2.72964872	0.20697957	0.04284054
RMSE	4.51726839	5.53069977	5.05432055	5.03412732	0.23496230	0.05520728
*R*-square	0.89421773	0.92943254	0.91146483	0.91236022	0.00822134	0.00006759
EVS	0.90510726	0.93987539	0.92421164	0.92471952	0.00666078	0.00004437

**Table 11:** Predictive performance evaluation profiles of TWT-QCF experiment for the testing phase with LHC-IVE.

Evaluation indicators	Minimum of indicators	Maximum of indicators	Mean of indicators	Median of indicators	Standard deviation of indicators	Variance of indicators
MAE	2.05089411	3.37652014	2.46878864	2.46178051	0.19748763	0.03900136
RMSE	3.47921884	6.20575030	4.49041956	4.47066517	0.28112794	0.07903292
*R*-square	0.89434556	0.96679048	0.94446434	0.94516681	0.00733756	0.00005384
EVS	0.90915484	0.96730075	0.94783112	0.94799915	0.00637982	0.00004070

## Data Availability

The data used to support the findings of this study are included within the article.
